# Deep Learning Approaches for Cyberbullying Detection and Classification on Social Media

**DOI:** 10.1155/2022/2163458

**Published:** 2022-06-11

**Authors:** Neelakandan S, Sridevi M, Saravanan Chandrasekaran, Murugeswari K, Aditya Kumar Singh Pundir, Sridevi R, T. Bheema Lingaiah

**Affiliations:** ^1^Department of CSE, R.M.K Engineering College, Kavaraipettai, India; ^2^Department of CSE, Anurag University, Telangana, India; ^3^Department of CSE, Saveetha School of Engineering, Saveetha Institute of Medical and Technical Sciences, Chennai, India; ^4^School of Computing Science and Engineering, VIT Bhopal University, Bhopal, India; ^5^Department of ECE, Arya College of Engineering and Information Technology, Kukas, Rajasthan, India; ^6^Department of CSE, K.Ramakrishnan College of Engineering, Samayapuram, India; ^7^School of Biomedical Engineering, Jimma Institute of Technology, Jimma, Ethiopia

## Abstract

As a result of the ease with which the internet and cell phones can be accessed, online social networks (OSN) and social media have seen a significant increase in popularity in recent years. Security and privacy, on the other hand, are the key concerns in online social networks and other social media platforms. On the other hand, cyberbullying (CB) is a serious problem that needs to be addressed on social media platforms. Known as cyberbullying (CB), it is defined as a repetitive, purposeful, and aggressive reaction performed by individuals through the use of information and communication technology (ICT) platforms such as social media platforms, the internet, and cell phones. It is made up of hate messages that are sent by e-mail, chat rooms, and social media platforms, which are accessed through computers and mobile phones. The detection and categorization of CB using deep learning (DL) models in social networks are, therefore, crucial in order to combat this trend. Feature subset selection with deep learning-based CB detection and categorization (FSSDL-CBDC) is a novel approach for social networks that combines deep learning with feature subset selection. The suggested FSSDL-CBDC technique consists of a number of phases, including preprocessing, feature selection, and classification, among others. Additionally, a binary coyote optimization (BCO)-based feature subset selection (BCO-FSS) technique is employed to select a subset of features that will increase classification performance by using the BCO algorithm. Additionally, the salp swarm algorithm (SSA) is used in conjunction with a deep belief network (DBN), which is known to as the SSA-DBN model, to detect and characterize cyberbullying in social media networks and other online environments. The development of the BCO-FSS and SSA-DBN models for the detection and classification of cyberbullying highlights the originality of the research. A large number of simulations were carried out to illustrate the superior classification performance of the proposed FSSDL-CBDC technique. The SSA-DBN model has exhibited superior accuracy to the other algorithms, with a 99.983 % accuracy rate. Overall, the experimental results revealed that the FSSDL-CBDC technique beats the other strategies in a number of different aspects.

## 1. Introduction

In recent years, people utilize virtual meeting platforms in their daily lives using global online social network (OSN) to facilitate communication. This network helps users for finding new friends and increases their connections around the world. Furthermore, sharing of data and opinions is the significant features of OSN [1–3]. In recent years, the rate of utilizing OSN has rapidly increased. With OSNs such as Facebook, Google+, LinkedIn, Twitter, VKontakte, Mixi, and Sina Weibo, a Japanese social network turned into the desired manner of transmission for billions of everyday active users. A user consumes maximal time for updating their content, interacting with primary user, and browsing others' account for finding particular data that are the major implication of social network website. OSN could remove the economical and geographical barriers among the users for sharing information and communication. In addition, OSN is highly beneficial to attain the objectives like amusement, education, search for jobs, etc. The popularity of OSN leads to high risks of an attack on the OSN users. Several OSN users expose their private data and that act as a proposal for the attacker to perform specific malicious activities [4, 5].

The current extensive nature of cyberbullying (CB) has enlarged the significance of its recognition. As per the survey, nearly 43% of the teenagers in the US alone have been stated to be the targets of CB at a certain point. CB is deliberated as a novel or electric method of conventional bullying. CB is determined as an aggressive, repeated, and intended response determined by an individual/group toward other individuals/groups, which is created using information and communication technology (ICT) methods like the internet, mobile phones, and social media [6]. The whole CB events are executed in internet broadcasting instead of in a physical system. The CB contains hate letters transferred by e-mails, social networking, and so on, via public/private computers/using private mobile phones. It is raised as a severe threat among the states. Current research displays the ratio as improved to be about 59% in the US. CB has a similar, when it is not a better, negative impact on the victim against conventional bullying, since the predators generally attack a victim on the aspect that an individual could not alter (viz., ethnicity, physical appearance, skin color, and religion), which leaves a deep and long-lasting effect on the victim. Occasionally, the related humiliations are sufficient for pushing the victim to self-infliction of suicide/harm.

A study in [7] displayed that suicide thoughts tend to rise among teenagers because of the disclosure of various types of CB. Although precautions are occupied, the redevelopment of victims of CB cases is challenging for society and families. Self-hate, dominance, isolation, and reaction to the socializing procedure lead to troubled and unhappy adults. Furthermore, this mental imbalance could alone make upcoming bullies. Among many problems, which create the recognition of CB in OSN is highly complicated, current advanced solution for detecting CB does not determine the possibility of bullying types in their detection method [8]. We specified the different kinds of CB, which could arise on the web, and it is not possible for assuming that a similar detection method would be effective in finding all types of bullying.

The main limitation present in the current detection system using CB study is the absence of input data. This study is traditionally executed on an available dataset/surveyed data, while the victim's/perpetrators are permitted for reporting the impression. Another issue with automatic CB identification is determining the most appropriate operation on CB material that takes into account the available studies in the CB detection region in order to achieve the goal of automatic detection accurately recognizing CB actions, which is another issue with automatic CB identification. It becomes more difficult to determine the actions as a result of this, and well-developed tools for combining the information via an autonomous decision technique are necessary [9]. To achieve the goal of automatic detection to precisely recognize CB actions, a CB detection zone was created. The automated decision-making is the process of making decisions without human intervention. Inferred data or digitally developed profiles can also be used to make these decisions. A preprogrammed algorithm and criteria may be used in an online loan decision or a recruitment aptitude examination. Administration heavily relies on automation. Automated systems can increase administrative decision-making consistency, correctness, and transparency, and enable new service delivery choices in the relevant areas and with suitable supervision. According to the findings of this study, machine learning was utilized to detect artificial CB material based on a number of psychological and common characteristics. The CB detection rate of this intelligent system has been reported to be lower, and it has been found to be mostly confined to a person writing a comment in the text [10]. The present research has stated that the consumption of user context in the event includes the history and features of user comments for improving the efficiency of CB classification or detection [11]. SSA with the DBN algorithm was used. Salp swarm algorithm (SSA) with deep belief network (DBN) is called as the SSA-DBN model. The SSA-DBN model is employed to detect and classify cyberbullying in social networks. For identifying suspicious attacks in a social, a salp swarm algorithm-based deep belief network is presented. As a result, the suggested chronological salp swarm algorithm-based deep belief network is constructed by fusing the chronological and salp swarm concepts. The fitness function, which accepts the minimal error vale as the optimal solution, reveals the optimal solution for detecting the incursion. The suggested approach tunes the weights appropriately in this case to produce an effective and optimal solution for identifying intruders.

This study presents a novel feature subset selection with DL-based CB detection and classification (FSSDL-CBDC) model on social networks. In addition, a binary coyote optimization-based feature subset selection (BCO-FSS) technique is applied to choose a set of features for enhanced classification efficiency. Moreover, the salp swarm algorithm (SSA) with deep belief network (DBN), called the SSA-DBN model, is working to detect and classify CB in social networks. Deep belief networks (DBNs) were created as a response to the issues that classic neural networks have with deep layered networks' training, such as slow learning, becoming stuck in local minima owing to poor parameter selection, and requiring much training datasets. The greedy algorithm is used to precondition deep belief networks—the design of the BCO-FSS and SSA-DBN models for CB detection and categorization procedure. To choose a set of features for improved classification efficiency, the binary coyote optimization-based feature subset selection (BCO-FSS) technique is used. To detect and classify CB in social networks, we combine the salp swarm algorithm (SSA) with a deep belief network (DBN) and dubbed the SSA-DBN model. BCO-FSS and SSA-DBN model development for CB detection and classification process demonstrates the effort's inventiveness. Furthermore, the utilization of the SSA to fine-tune the hyperparameter of the DBN model resulted in enhanced outcomes over the traditional DBN model. The BCO technique is applied to choose a set of features for enhanced classification efficiency, and the SSA is employed to detect and classify cyberbullying in social networks. For the exploratory better detection presentation of the proposed FSSDL-CBDC method, a comprehensive range of simulations was performed on a benchmark dataset.

## 2. Related Works

This section reviews the recently developed automated CB classification models on social networks. Yuvaraj et al. [12] integrate the classification and feature extraction engine. The classification engine utilizing ANN categorizes the result, and it is given by a calculation scheme that either penalizes/rewards the categorized output. DRL performs the calculations, which increases the efficiency of classification. In their study, Mahbub et al. [13] investigate the impact of predatory approach words on CB detection and present a method for generating a vocabulary of predatory approach phrases. This study brings together findings from investigations of convicted criminals' chat logs in order to develop a lexicon of sexual approach terms for use in the future. Through the examination of data from a variety of social networks, the research establishes the relevance of this dictionary of approach terms in detecting online predatory behavior via machine learning methodologies. The variety of contents available on different social media sites are demonstrated by this example.

Talpur and O'Sullivan [14] created a supervised machine learning strategy for detecting CB and categorizing its severity on Twitter, which they published in Nature. The text classification engine created by Yuvaraj et al. [15] that preprocesses tweets, eliminates noisy data and other background information, extracts the desired features, and categorizes without overfitting the data is described in detail below. This research advances a novel DDT strategy that processes input components by utilizing the DNN hidden layer as tree nodes, as demonstrated in previous research. Chia et al. [16] use feature engineering and machine learning approaches to explore the use of irony and sarcasm on social media platforms. To begin, they define and assess the definitions of sarcasm and irony by looking at a large number of research studies that are focused on the contexts in which they are used. Subsequently, a comparison of numerous classification approaches with a few widely used classification schemes for the text classification process is carried out following the initial research. A variety of methods of data preprocessing were examined and compared in the following research.

In Murnion et al. [17], an automated data collection scheme is proposed that always gathers game chat data from the common online multiple player games. The data have been combined and collected using other data regarding the companies from the presented connected data service. It presented a scoring system for enabling the detection of CB depending upon this study. The organization of the gathered data was executed by humble feature recognition with SQL database enquiries and related with classifications from the AI-based sentimentality text analysis services, which have currently turned into presented and automatically classified data utilizing custom-built classification user.

Bu and Cho [18] proposed an ensemble technique of the 2 DL methods: first is character-level CNN that takes lower-level syntactic data from the series of characters and strong to the noise by the TL method. Next is word-level LRCN that takes higher-level semantic data from the series of words, accompanying the CNN module. Kumari and Singh [19] extract integrated features of text and images for identifying distinct events of CB. They utilize a pretrained VGG-16 network and CNN for extracting the features from text and images, correspondingly. These features are additionally improved by GA for increasing the performance of the entire system. Al-Garadi et al. conducted an in-depth research on cyberbullying prediction models on social media and identified several unresolved issues, including the prediction of cyberbullying intensity, human data features, and language dynamics. Numerous studies examine various machine learning options for detecting cyberbullying. Hosseinmardi et al. investigate the detection of cyberbullying episodes on the social media platform Instagram. They employ naive Bayes and SVM classifiers, the latter of which achieves the highest performance by combining multimodal text and image information, and media session data. Several other studies concentrate on the characteristics believed to be associated with cyberbullying, such as analyzing the social network structure of users, combining text and picture analysis techniques, profanity features, sentiment analysis, or geographical features, among others.

## 3. The Proposed Model

As illustrated in Figure 1, the operating principle of the FSSDL-CBDC approach is described. Several steps are required for the proposed FSSDL-CBDC technique to be effective, including preprocessing, feature selection using BCO-FSS, and classification using SSA-DBN. The FSSDL-CBDC technique was used. A variety of simulations were run to demonstrate the proposed FSSDL-CBDC technique's improved classification performance. Cyberbullying is a pernicious form of online abuse of authority that has malicious consequences. It takes on a variety of formats, and in the majority of social media platforms, it is in textual format. Intelligent systems are required to automatically detect such situations. Deep learning-based models have made their way into the detection of cyberbullying occurrences, claiming to be able to overcome the limits of conventional models and significantly enhance detection performance. The activities of these processes are described in greater detail in the following sections.

### 3.1. Preprocessing

During preprocessing, a lexical normalization technique is employed, which makes use of different elements for cleaning the input data. It also transforms the numerical parameters to the corresponding textual data. In addition, a spell corrector tool is used to eradicate the outbound vocabulary words. In addition, the repetitive or missing parameters are removed involving spelling mistakes, incorrect punctuation marks, and so on.

### 3.2. Design of the BCO-FSS Technique

Once the input social network data are preprocessed, they are fed into the BCO-FSS technique. The COA is a strong populace-based method projected lately by Juliano and Leandro [20]. This method draws stimulation from the common behaviors of *Canis latrans* species that live mostly in the NA. Because of its exclusive form, the COA could be categorized as evolutionary heuristics and swarm intelligence (SI). The coyote's population is separated to *N*_*p*_ packs, and *N*_*c*_ coyotes for each pack. The amount of coyotes in apiece pack is thought to be constant and equal. As a result, the populace size may be calculated by multiplying *N*_*p*_ and *N*_*c*_. Every coyote's social status denotes a potential solution $\overset{⟶}{\text{x}}$ to the optimization issue. In this case, the communal situation of c^th^ coyote in p^th^ packet at t^th^ time may be described as follows:

(1) $$\begin{array}{c} {\text{soc}}_{c}^{p,t}=\overset{⟶}{x}=\left(x_{1},x_{2},\ldots ,x_{D}\right), \end{array}$$

where *D* represents the amount of dimension in the search space. Initially, a population of *N*_*p*_ × *N*_*c*_ coyote is arbitrarily initiated within the predetermined search space as follows:

(2) $$\begin{array}{c} {\text{soc}}_{c\dot{j}}^{p,t}={\text{lb}}_{j}+r_{j}\cdot \left({\text{ub}}_{j}-{\text{lb}}_{j}\right), \end{array}$$

where lb and ub denote lower and upper bounds of *j*^th^ decision variable, correspondingly. *r*_*j*_ represents real number arbitrarily created among zero and one, succeeding uniform distributions. Then, the adaption of coyotes to their corresponding social condition is estimated by the following:

(3) $$\begin{array}{c} {\text{fit}}_{c}^{p,t}=f\left({\text{soc}}_{c}^{p,t}\right). \end{array}$$

As mentioned, the coyotes tend to leave their present pack for leading a lonely life or join other packs. The exclusion of coyote from its pack shadows a likelihood *P*_*e*_, which differs based on the pack size as follows:

(4) $$\begin{array}{c} P_{e}=0.005\cdot N_{c}^{2}. \end{array}$$

This method improves population range by stimulating a global interchange of data between the coyote packs. As *P*_*e*_ goes beyond one for *N*_c_$\geq \sqrt{200}$, the COA limits the maximal amount of coyotes for each pack to fourteen [21]. In every pack, the coyote is optimally familiarized with the atmosphere and is allocated as alpha. For the minimization problem, the alpha is given as

(5) $$\begin{array}{c} {\text{alpha}}^{p,t}=\left\{{\text{soc}}_{c}^{p,t}|{\text{arg}}_{c}=\left\{1,2,\ldots ,N_{c}\right\}\text{min }f\left({\text{soc}}_{c}^{p,t}\right)\right\}. \end{array}$$

With the consideration of clear indications of the SI in coyotes, the COA assumes all the coyotes' share their social condition with the remaining packs for improving the pack's survivability. Regarding this, the traditional tendency of a pack is determined according to the data given its member, ciz.,

(6) $$\begin{array}{c} {\text{cult}}_{j}^{p,t}=\left\{\begin{array}{cc} O_{\left(Nc+1\right)/2}^{p,t} & N_{c}\text{ is odd}\\ \frac{O_{\left(Nc/2\right),j}^{p,t}+O_{\left(Nc+1\right)/2,j}^{p,t}}{2} & \text{otherwise} \end{array}\right), \end{array}$$

where *O*^*p*,*t*^ represents hierarchical communal condition of the prairie wolf within *p*^th^ pack at *t*^th^ time, for *j*=1,2,…, *D*. In this method, the traditional propensity of every pack is calculated as the middle of the combined communal condition within the carton. For modeling the two main organic proceedings of the coyote, namely, birth and death, the ages of every coyote are deliberated, age ∈ N. The birth of novel coyotes is defined by the combination among the communal circumstances of the two arbitrary parental coyotes from similar packs, and the effect of the environmental factor *R*_*j*_,

(7) $$\begin{array}{c} {\text{pup}}_{j}^{p,t}=\left\{\begin{array}{cc} {\text{soc}}_{r1,j}^{p,t}, & r\text{ and }j<P_{a}\text{ or }j=j_{1}\\ {\text{soc}}_{r2,j}^{p,t}, & r\text{ and}<P_{s}+P_{a}\text{ or }j=j_{2}\\ R_{j},\; & \text{otherwise} \end{array}\right), \end{array}$$

where soc_*r*1,*j*_^*p*,*t*^ and soc_*r*2,*j*_^*p*,*t*^ denote arbitrary coyote from the *p*^th^ pack, and *j*_1_ and *j*_2_ denote two arbitrary dimensions of the search space. Alternatively, *P*_*s*_ and *P*_*a*_ denote scatter and relationship likelihoods, correspondingly. *R*_*j*_ denotes arbitrarily created vector within the bounds of *j*^th^ dimension, and *r* and_*j*_ denotes uniformly arbitrary amounts in zero and one. The scatter and relationship likelihoods have a substantial impact on the composition and diversity of the coyote's pack. It is given by the following:

(8) $$\begin{array}{c} P_{s}=\frac{1}{D},\\ P_{a}=\frac{\left(1-P_{s}\right)}{2}. \end{array}$$

Based on this, the coyote's pup has around 10% chance of death at birth. Moreover, the death risk of every coyote increases with age. Thus, the COA designs the coyote's survivability depending upon a simple method, whereas *ω* and *φ* denote set of coyotes fewer adapted to the atmosphere (viz. worst fitness value) compared to pup and size of the groups, correspondingly.

Additionally, the COA represents the traditional communication among the coyotes in the pack using *δ*_1_ and *δ*_2_. The previous denotes the effect of alpha on an arbitrary coyote cr_1_, where the later indicates the effect of the traditional tendency of the pack on other arbitrary coyotes *cr*_2_. The cr_1_ and cr_2_ are chosen after a uniformly distributed likelihood. Therefore, *δ*_1_ and *δ*_2_ are given by

(9) $$\begin{array}{c} \delta_{1}={\text{alpha}}^{p,t}-{\text{soc}}_{cr1}^{p,t}, \end{array}$$

 

(10) $$\begin{array}{c} \delta_{2}={\text{cult}}^{p,t}-{\text{soc}}_{cr2}^{p,t}. \end{array}$$

The social condition of the coyote is inclined by the alpha, and other members of the pack will be upgraded using

(11) $$\begin{array}{c} \text{new }{\text{soc}}_{c}^{p,t}={\text{soc}}_{c}^{p,t}+r_{1}\cdot \delta_{1}+r_{2}\cdot \delta_{2}, \end{array}$$

where *r*_1_ and *r*_2_ are random values. The coyotes of new social conditions are assessed using

(12) $$\begin{array}{c} \text{new }{\text{fit}}_{c}^{p,t}=f\left(\text{new}-{\text{soc}}_{c}^{p,t}\right). \end{array}$$

The coyotes' general fitness will either increase or remain the same, but it will never deteriorate.

(13) $$\begin{array}{c} {\text{soc}}_{c}^{p,t+1}=\left\{\begin{array}{cc} {\text{new}}_{-}{\text{soc}}_{c}^{p,t} & \text{if new}-{\text{fit}}_{c}^{p,t}<{\text{fit}}_{c}^{p,t}\\ {\text{soc}}_{c}^{p,t} & \text{otherwise} \end{array}\right). \end{array}$$

Additional features could inhibit the learning procedure. The FS could authenticate the significance of the features, which create a dataset, and removing these does not assist in a positive manner. The selected features using an FS method could be denoted as N-sized vector, whereas N denotes the overall number of features in a dataset, whereas every position of the vector could consider the values as zero/one, whereas zero denotes features that were not chosen as also one signifies features that were chosen. The transfer purpose technique determines the likelihood of altering a position vector component from zero to one and conversely in an efficient and simple manner, and hence, the binarization method is the utilized most, particularly for the FS problem [22]. Based on this, a transfer function considerably affects the efficiency of the FS methods in seeking an optimal set of features, concerning the local optimal prevention and the balance between exploitation and exploration, and thus, it is a significant role in the binary version of metaheuristics. In the BCOA, the constraint of the social conditions of coyotes for the binary values by a V-shaped transfer function is defined by equation (14) as follows:

(14) $$\begin{array}{c} V\left(\text{new}\_{\text{soc}}_{c}^{p,t}\right)=\left|\frac{\text{new}\_{\text{soc}}_{c}^{p,t}}{\sqrt{1+{\left(\text{new}\_{\text{soc}}_{c}^{p,t}\right)}^{2}}}\right|, \end{array}$$

where new_soc_*c*_^*p*,*t*^ relates to the upgraded social condition vector existing, considering continuous values.

### 3.3. Algorithmic Design of the SSA-DBN Technique

Once the subsets have been feature-reduced, they are fed into the SSA-DBN model, which is then utilized to complete the classification assignment. This is accomplished through the use of the DBN model, which generates feature vectors that are then classified using the softmax layer. By picking hyperparameter values in the most optimal method, the SSA is used to improve the detection performance of a DBN model, whereas the SSA is used to improve its detection performance.

#### 3.3.1. Architecture of DBN

Since DBN contains multiple hidden levels and countless hidden units within each of those layers, it is considered a member of the DNN family. The standard DBN technique is similar to the RBM technique in that it includes an output layer. Additionally, the DBN achieves its outcomes using a strong, greedy unsupervised learning technique to train RMB, and a supervised fine-tuning mechanism that adjusts the scheme using labeled data. The RBM is composed of two types of layers: visible and buried layers coupled with undirected weights. When RBMs are stacked in DBN, the RBM's hidden layer is chosen to be the visible layer of the subsequent RBM. This is because the RBM's hidden layer provides information about the subsequent RBM. RMB's variable sets are defined as =(*w*, *b*, *a*), where *w* ij is the weight difference between *v* I and *h* j. The bias layers *b* I and a *j* must be identified.

Figure 2 displays the framework of DBN. The RBM defines equivalent energy as described as follows:

(15) $$\begin{array}{c} E\left(v,h|\theta \right)=-\underset{i}{\sum }b_{i}v_{i}-\underset{j}{\sum }a_{j}h_{j}-\underset{i}{\sum }\underset{j}{\sum }w_{ij}v_{i}h_{j}. \end{array}$$

The joint likelihood distribution of *v* and *h* is defined below as follows:

(16) $$\begin{array}{c} p\left(v,h|\theta \right)=\frac{\exp\left(-E\left(v,h|\theta \right)\right)}{\sum_{v,h}\exp\left(-E\left(v,h|\theta \right)\right)}. \end{array}$$

Here, the marginal likelihood distribution of *v* is established by

(17) $$\begin{array}{c} p\left(v|\theta \right)=\;\frac{\sum_{h}\exp\left(-E\left(v,h|\theta \right)\right)}{\sum_{v,h}\exp\left(-E\left(v,h|\theta \right)\right)}. \end{array}$$

To gain an optimum *θ* value for a solitary data vector *v*, the incline of log probability approximation is evaluated by [23]the following:

(18) $$\begin{array}{c} \frac{\partial \;\log p\left(v|\theta \right)}{\partial w_{ij}}=v_{i}h_{j\text{ data}}-v_{i}h_{j\text{ model}},\\ \frac{\partial \;\log p\left(v|\theta \right)}{\partial a_{j}}=h_{j\text{ data}}-h_{j\text{ model}},\\ \frac{\partial \;\log p\left(v|\theta \right)}{\partial b_{i}}=v_{i\text{ data}}-v_{i\text{ model}}. \end{array}$$

Here, 〈•〉 denotes expectation using the delivery of a specific subscript. Because of the lack of influences between units within the same layer, 〈∙〉_data suggests that it may be obtained by measuring the conditional likelihood distribution by measuring the provisional likelihood delivery by

(19) $$\begin{array}{c} p\left(h_{j}|v,\;\theta \right)=\frac{1}{1+\text{exp}\left(-\sum_{j}w_{ij}v_{i}-a_{j}\right)},\\ p\left({\text{v}}_{i}|\text{h},\;\theta \right)=\frac{1}{1+\text{exp}\left(-\sum_{j}w_{ij}h_{j}-b_{i}\right)}. \end{array}$$

Due to the shape of the activation function, it is referred to as a sigmoid function. Contrastive divergence can be regarded of as a learning technique that approximates maximum likelihood. It calculates the divergence/differences between the positive phase (energy of first encoding) and the negative phase (energy of second encoding) (energy of the last encoding). To reduce the variation of two Kullback-Leibler divergences through renovation, the contrastive divergence (CD) learning module is used in the case of _model (KL). To begin, the CD learning is more efficient than Gibbs sampling in real-world applications and requires less processing time. Thus, weights in the DBN layer are taught using unlabeled data by unsupervised algorithms that are both fast and greedy in their information search. For predictions, the DBN uses the supervised layer to fine-tune the learned features using labeled data from the training set. The fully connected (FC) layer is now the top layer, and the layers beneath it are activated using the sigmoid activation function.

#### 3.3.2. Overview of SSA

The SSA is a novel SI method, which was established lately by [24]. The main concept behindhand in the SSA operator is that they simulate the swarming behavior of salp in deep oceans. Salp belonged to the species of Salpidae and contain transparent barrel-shaped bodies. They are related to jellyfishes in their tissue and motion. Moreover, they shift as the water is driven by the body as a force to move onward. The salp provides a novel 160 forms of swarm called a slapping chain while directing in the ocean. The salp chain behavior was numerically modeled by separating the population into groups depending upon leader and follower. The front of the chain is deliberated as the led 1 when the remaining salps are called as followers. The leader's part is to direct the swarm of salp, and all the followers follow the previous one. Related to the other SI techniques, the procedure of SSA imitates by initiating an arbitrary population of salp and later evaluates the fitness for every salp [25]. The slap with an optimal best fitness value is represented as a front-runner salp, whereas an additional slap is symbolized as a follower. The salp swarm algorithm (SSA) is a new stochastic algorithm inspired by salps' navigational and foraging abilities. However, higher dimension problems show a poor convergence rate for classical SSA. The SSA lacks exploration and exploitation, resulting in inefficient convergence. A salp's best fitness is found by exploring and exploiting the search space. The leader's salp location is modified based on the distance between the salp and food supply. The optimal performing slaps are represented as a food source to be chased using a salp chain. For updating the location of the slap chain, two major stages are determined: leader and follower phases.

The location of the leader is upgraded by equation (20) as follows:

(20) $$\begin{array}{c} X_{j}^{1}=\left\{\begin{array}{c} X_{{\text{Best}}_{j}}+c_{1}\left(\left(ub_{j}-lb_{j}\right)c_{2}+lb_{j}\right)\text{ if }c_{3}\geq 0.5,\\ X_{{\text{Best}}_{j}}-c_{1}\left(\left(ub_{j}-lb_{j}\right)c_{2}+lb_{j}\right)\text{else,} \end{array}\right) \end{array}$$

where *X*_*j*_^1^ and *X*_Best_*j*__ represent novel location of leader and food source in *jth* dimension, and ub_*j*_ and lb_*j*_ represent upper and lower bounds of *j*^th^ dimension, correspondingly. *c*_2_ and *c*_3_ denote arbitrarily created amounts in the range zero and one . The variable *c*_1_ presents an important aspect in the SSA that controls the balance between exploration and exploitation. Moreover, *c*_1_ gradually decreases by iteration as displayed in the following equation (21):

(21) $$\begin{array}{c} c_{1}=2e^{-{\left(4t/T\right)}^{2}}, \end{array}$$

where *t* specifies present iteration, and *T* denotes maximal amount of 152 iterations.  Figure 3 exemplifies the flowchart of the SSA. For updating the location of follower, novel idea is presented where 185 is depending upon Newton's law of movement as in equation (22).

(22) $$\begin{array}{c} X_{j}^{i}=\frac{1}{2}gt^{2}+w_{0}t,\;i\geq 2, \end{array}$$

where *X*_*j*_^*i*^ denotes location of *i*^th^ follower salp in *j*^th^ dimension. In the optimization procedure, the time *t* corresponds to the present iteration, 188, whereas *g* and *w*_0_ indicate velocity and acceleration, correspondingly. In equation (22), the early speed *w*_0_ is set to zero and the inconsistency is set 190 to one (△*t*=1); thus, the upgrading procedure of follower is equated in 191 equation (23).

(23) $$\begin{array}{c} X_{j}^{i}j=\frac{1}{2}\left(X_{j}^{i}+X_{j}^{i-1}\right). \end{array}$$

#### 3.3.3. Parameter Optimization of DBN Using SSA

For optimally regulating the hyperparameters of the DBN model, the SSA is used and the detailed working is provided in the following. The training process of the DBN model takes place using a fitness function [26–30]. In addition, 10‐fold cross‐validation (CV) process is utilized to evaluate the FF. Under 10‐fold CV, the training dataset is randomly subdivided into a collection of ten equally exclusive subsets of nearly equal sizes, where nine subsets are used to train the data, and the remaining one is applied to test the data. These processes are repeated for a set of 10 iterations in such a way that each subset can be used to test the model. The FF is denoted as 1‐CA_validation_ of the 10‐fold CV model in the training data, as defined in equation (24). Also, a solution with maximum CA_validation_ leads to minimal fitness value [31–33].

(24) $$\begin{array}{c} \text{Fitness}=1-CA_{\text{validation}},\\ {\text{CA}}_{\text{validation}}=1-\frac{1}{10}\overset{10}{\underset{i=1}{\sum }}\left|\frac{y_{c}}{y_{c}+y_{f}}\right|\times 100, \end{array}$$

where y_c_ and y_f_ indicate the true and false organization count. Finally, the hyperparameter involved in the DBN model is optimally picked up by the SSA, and also, the performance of classification gets improved.

## 4. Performance Evaluation

In this section, we validate the proposed model performance under several aspects.  Table 1 investigates the performance of the feature selection techniques in terms of classification accuracy under different sets of training data and varying number of residuals [34, 35].  Figure 4 examines the result analysis of different feature selection techniques in terms of classification accuracy on 60% of training data. From the figure, it is depicted that the BCO-FSS model is found to be an effective method and it leads to maximum classification accuracy. For instance, under 200 residuals, the proposed BCO-FSS technique has accomplished a higher classification accuracy of 28.61%, whereas Pearson's correlation, chi-squared, and information gain techniques have resulted in a lower classification accuracy of 28.61%, 27.10%, and 25.18%, respectively.

Moreover, under 1000 residuals, the BCO-FSS technique has obtained an increased classification accuracy of 37.80%, whereas Pearson's correlation, chi-squared, and information gain techniques have attained a decreased classification accuracy of 34.78%, 32.68%, and 29.46%, respectively.

Figure 5 inspects the outcome analysis of different feature selection approaches with respect to classification accuracy on 75% of training data. From the figure, it can show that the BCO-FSS method is found to be an effective technique and it leads to maximal classification accuracy. For instance, under 200 residuals, the presented BCO-FSS manner has accomplished a higher classification accuracy of 43.24%, whereas Pearson's correlation, chi-squared, and information gain methods have resulted in a lesser classification accuracy of 40.39%, 36.26%, and 34.65%, correspondingly. Furthermore, under 1000 residuals, the BCO-FSS technique has gained an improved classification accuracy of 66.26%, whereas Pearson's correlation, chi-squared, and information gain techniques have achieved a reduced classification accuracy of 60.07%, 55.47%, and 52.19%, correspondingly.

Figure 6 investigates the result analysis of different feature selection methods in terms of classification accuracy on 90% of training data. From the figure, it can be stated that the BCO-FSS manner is initiated to be an effective approach and it leads to higher classification accuracy. For sample, under 200 residuals, the projected BCO-FSS method has talented a larger classification accuracy of 47.44%, while Pearson's correlation, chi-squared, and information gain techniques have resulted in a lower classification accuracy of 43.88%, 39.55%, and 33.29%, correspondingly. Also, under 1000 residuals, the BCO-FSS technique has attained a maximum classification accuracy of 74.18%, whereas Pearson's correlation, chi-squared, and information gain techniques have gained a lesser classification accuracy of 69.60%, 64.51%, and 59.61%, correspondingly.

If fewer than 60% of the training data are available, the suggested SSA-DBN model is compared to existing techniques in Table 2.  Figure 7 displays an overview of the SSA-DBN model's sensitivity and specificity studies, which were conducted using the comparable methodologies. The LR model performed worse than the LR model, as seen in the figure, with a sensitivity of 74.335 % and a specificity of 75.025 %, respectively. It was expected that the RF model would produce a little better result, with a sensitivity of 74.825 % and a specificity of 78.196 %, and the RF model did so. Furthermore, the SVM model displayed significantly improved performance, with a sensitivity of 76.506 % and a specificity of 83.708 %, respectively, compared to the baseline model. The ANN model also generated moderate results, with a sensitivity of 76.976 % and a specificity of 84.719 %, respectively, for the sensitivity and specificity tests. Aside from that, the NB model provided a tolerable outcome, as evidenced by its sensitivity of 80.657 % and specificity of 73.475 %, among other statistics. Additionally, the ANN-DRL model must yield competitive outcomes with 83.598 percent% sensitivity and 85.129 % specificity in order to be considered successful. But the proposed SSA-DBN model outperformed the competition, with sensitivity and specificity values of 85.728 % and 88.728 %, respectively, in the study.

Figure 8 offers a comparative analysis of the SSA-DBN with other classifiers in terms of accuracy, F-measure, and G-mean. The obtained results illustrated that the NB and LR models have attained a lower accuracy of 61.821 and 69.023, respectively. Next, the RF and SVM models have showcased moderately closer presentation with the correctness of 71.814% and 77.236%, respectively. In addition, the ANN and ANN-DRL techniques have showcased reasonable consequences with the correctness of 80.897% and 85.369%, correspondingly. However, the SSA-DBN perfect has outperformed the other methods with a maximum accuracy of 88.473%.

On the following page, you will find a quick comparison of the given SSA-DBN approach to alternative strategies that use less than 75 % of the training data.  Figure 9 displays a detailed sensitivity and specificity evaluation of the SSA-DBN model, which was carried out utilizing comparative methodology. In this study, we discovered that the NB approach had lower sensitivity than the other methods (68.593 %) but greater specificity than the other methods (98.093 %). Additionally, the LR strategy produced somewhat better outcomes, with a sensitivity of 69.583 % and a specificity of 98.583 %, respectively, compared to the LR approach. Afterward, the RF algorithm displayed significantly improved performance, with a sensitivity of 70.074 % and a specificity of 98.513 %, respectively, compared to the baseline algorithm. The SVM model also performed well in terms of sensitivity and specificity, scoring 70.394 % and 98.663 %, respectively, for mild outcomes in the study. As an additional benefit of using the artificial neural network model, a tolerable outcome was achieved with a sensitivity of 72.614 % and a specificity of 98.553 %. At the same time, the ANN-DRL model aimed to exhibit competitive outcomes with 73.315 % compassion and 98.353 % specificity while also attempting to demonstrate competitive outcomes. However, the accessible SSA-DBN practice obtained optimal performance, with a compassion rate of 79.063 % and a specificity rate of 98.976 %, respectively, compared to the other practices tested in Table 3.

Figure 10 provides a comparative analysis of the SSA-DBN with other classifiers with respect to accuracy, F-measure, and G-mean. The attained outcomes showcased that the NB and RF methods have attained a lower accuracy of 96.743 and 96.993, correspondingly. Next, the SVM and LR techniques have depicted moderately closer performance with the accuracy of 97.003% and 97.063%, correspondingly. Also, the ANN and ANN-DRL techniques have exhibited reasonable consequences with the correctness of 97.553% and 97.313%, respectively. However, the SSA-DBN perfect has outperformed the other techniques with a maximal accuracy of 98.362%.

With less than 90 % of the training data, the anticipated SSA-DBN model's performance is compared to the performance of other techniques, which is presented in detail in Table 4. According to the comparison methodologies used in this work, the SSA-DBN model's sensitivity and specificity were briefly evaluated (Figure 11). In the figure, it can be seen that the LR technique fared poorer than the other approaches, with a sensitivity of 92.766 % and a specificity of 99.583 %. Although the NB technique produced a little better results than expected (sensitivity 92.796 % and specificity 99.673 %), it did so in a more consistent manner. A similar improvement in performance was seen in the RF model, which had a sensitivity of 93.537 % and a specificity of 99.773 % when compared to the baseline model. The SVM model also showed moderate results, with a sensitivity of 93.697 % and a specificity of 99.803 %, respectively, according to the results of the study. In addition, the ANN model provided a tolerable outcome, with a sensitivity of 94.387 % and a specificity of 99.733 %, according to the results. As part of this effort, the ANN-DRL approach aimed to simultaneously exhibit competitive outcomes. The method's sensitivity and specificity were both 99.873 %, indicating that it was successful in demonstrating competitive outcomes. The new SSA-DBN model, on the other hand, outperformed the prior model, with sensitivity and specificity values of 96.037 and 99.997 %, respectively, in comparison.

Figure 12 gives a comparative analysis of the SSA-DBN with other classifiers in terms of accuracy, F-measure, and G-mean. The attained results demonstrated that the NB and RF approaches have attained a lower accuracy of 99.503 and 99.623, respectively. In addition, the LR and SVM copies have showcased abstemiously closer presentation with the correctness of 99.633% and 99.673%, correspondingly. At the same time, the ANN and ANN-DRL manners have showcased reasonable consequences with the correctness of 99.563% and 99.703%, congruently. However, the SSA-DBN perfect has demonstrated the other algorithms with a higher accuracy of 99.983%.

## 5. Conclusions

In this post, we will describe a novel FSSDL-CBDC technique for detecting and classifying cyberbullying in social media, and how to apply it. The suggested FSSDL-CBDC technique consists of a number of phases, including preprocessing, feature selection, and classification, among others. Additionally, by creating the BCO-FSS approach to choose the optimal collection of features from the preprocessed data, the overall classification results are significantly enhanced. Figure 1 shows the BCO-FSS technique design. The SSA-DBN model receives and classifies the feature-reduced subset in the same time frame as the other models. When compared to the classic DBN model, the usage of the SSA to fine-tune the DBN model's hyperparameter resulted in improved outcomes when using the SSA. A large number of simulations on a benchmark dataset were carried out in order to assess the increased detection performance of the proposed FSSDL-CBDC technique, which was found to be effective. When compared to other state-of-the-art approaches, the simulation results revealed that the FSSDL-CBDC strategy performed significantly better in classification than the others. In the future, the performance of the FSSDL-CBDC technique may be enhanced by including outlier identification and feature reduction techniques in the algorithm. Unsupervised feature selection (FS) for outlier detection (OD) in streaming data (SD) for fields such as intrusion detection and network security, which are increasingly challenged with large amounts of high-dimensional data that must be analyzed in near real time.

## Figures and Tables

**Figure 1:** Working process of the FSSDL-CBDC model.

**Figure 2:** DBN structure.

**Figure 3:** Flowchart of SSA.

**Figure 4:** Classification accuracy analysis of the BCO-FSS model on 60% of training data.

**Figure 5:** Classification accuracy analysis of the BCO-FSS model on 75% of training data.

**Figure 6:** Classification accuracy analysis of the BCO-FSS model on 90% of training data.

**Figure 7:** Sensitivity and specificity analysis of the SSA-DBN model on 60% training data.

**Figure 8:** Comparative analysis of the SSA-DBN model on 60% training data.

**Figure 9:** Sensitivity and specificity analysis of the SSA-DBN model on 75% training data.

**Figure 10:** Comparative analysis of the SSA-DBN model on 75% training data.

**Figure 11:** Compassion and specificity analysis of the SSA-DBN model on 90% of training data.

**Figure 12:** Comparative analysis of the SSA-DBN model on 90% training data.

**Table 1:** Consequences of existing with future feature assortment methods on various training data size.

Classification accuracy on 60% training data				
Residuals	BCO-FSS	Pearson correlation	Chi-squared	Information gain
200	28.61	27.10	25.18	23.21
400	31.87	30.47	28.26	26.54
600	33.09	31.23	29.43	27.41
800	35.30	33.15	31.29	28.97
1000	37.80	34.78	32.68	29.46

Classification accuracy on 75% training data				
Residuals	BCO-FSS	Pearson correlation	Chi-squared	Information gain

200	43.24	40.39	36.26	34.65
400	53.24	50.07	44.36	41.84
600	55.94	51.66	47.85	43.75
800	61.02	56.10	51.66	48.06
1000	66.26	60.07	55.47	52.19

Classification accuracy on 90% training data				
Residuals	BCO-FSS	Pearson correlation	Chi-squared	Information gain

200	47.44	43.88	39.55	33.29
400	61.45	56.10	49.23	44.62
600	66.80	57.88	45.92	40.90
800	67.82	60.69	52.28	48.47
1000	74.18	69.60	64.51	59.61

**Table 2:** Results of existing with the proposed SSA-DBN on predicting cyberbullying with 60% training data.

Measures	NB	LR	RF	SVM	ANN	ANN-DRL	SSA-DBN
Accuracy	61.821	69.023	71.814	77.236	80.897	85.369	88.473
F-measure	72.674	72.965	73.045	73.325	77.876	83.588	86.901
G-mean	73.115	73.065	74.895	76.856	79.427	82.008	84.371
Sensitivity	80.657	74.335	74.825	76.506	76.976	83.598	85.728
Speciﬁcity	73.475	75.025	78.196	83.708	84.719	85.129	88.728

**Table 3:** Results of existing with proposed SSA-DNN on predicting the cyberbullying with 75% training data.

Measures	NB	LR	RF	SVM	ANN	ANN-DRL	SSA-DBN
Accuracy	96.743	97.063	96.993	97.003	97.553	97.313	98.362
F-measure	61.281	62.901	63.491	63.891	65.242	65.552	70.466
G-mean	82.238	82.498	83.388	83.468	84.499	85.189	88.471
Sensitivity	68.593	69.583	70.074	70.394	72.614	73.315	79.063
Speciﬁcity	98.093	98.583	98.513	98.663	98.553	98.353	98.976

**Table 4:** Results of existing with the proposed SSA-DNN on predicting cyberbullying with 90% of training data.

Measures	NB	LR	RF	SVM	ANN	ANN-DRL	SSA-DBN
Accuracy	99.503	99.633	99.623	99.673	99.563	99.703	99.983
F-measure	88.071	88.191	90.213	90.063	91.454	91.455	94.378
G-mean	96.299	96.269	96.530	96.640	97.030	97.000	98.361
Sensitivity	92.796	92.766	93.537	93.697	94.387	94.418	96.037
Speciﬁcity	99.673	99.583	99.773	99.803	99.733	99.873	99.997

## Data Availability

This article contains all of the data.
